# Construction of Sports Nutrition Dynamic Intervention Mechanism Based on the Improvement of College Students' Physical Health

**DOI:** 10.1155/2022/2417523

**Published:** 2022-08-02

**Authors:** Dongsheng Wang, Baoping Chen

**Affiliations:** ^1^Sports Department, Henan College of Industry & Information Technology, Jiaozuo, 454000 Henan, China; ^2^College of Physical Education, Yuxi Normal University, Yuxi, 653100 Yunnan, China

## Abstract

Exercise can improve people's physical health and strengthen their body bones. But the physique of college students is generally too poor. The enhancement of College Students' physique cannot be completed in a day. This study aims to explore the best sports nutrition intervention scheme for strengthening college students' physique from the construction of sports nutrition dynamic intervention mechanism, so as to provide theoretical reference for public physical education teaching and students' independent exercise. In this study, 100 full-time associate students in our university were selected as the research objects. Before the experiment, the subjects' body shape, body function, and physical quality were tested. Based on the random mathematical method, the full-time associate students were randomly divided into four groups: control group, exercise intervention group, nutrition intervention group, and sports nutrition intervention group, with 25 people in each group. After the experiment, the body shape, body function, and physical quality of the four groups were tested. The results show that exercise and nutrition intervention have little effect on college students' height, but have great influence on body mass index, vital capacity and 800 meter running. Especially after the experiment, the vital capacity of the exercise group and the sports nutrition group increased by nearly 250 ml and 500 ml, respectively, and the 800 m running time increased by nearly 10 s and 18 s, respectively. Strengthening exercise and increasing nutritional intake can effectively improve the institutional health of college students.

## 1. Introduction

### 1.1. Background and Significance

At present, the national physical health monitoring results released by the ministry of education show that the physique level of full-time associate students in China has shown a downward trend in the past decade. According to the analysis of the National College Students' physical health status released by the Ministry of education in 2018, while the height and weight of Chinese college students are increasing, their sensitivity, explosive power, endurance, strength, and other manifestations are on the decline trend, especially that the decline of muscle strength and endurance is very obvious. Nutrition of students' diet is very important for physical health. As the future of the motherland, full-time associate students shoulder the important task of building the motherland. They are the driving force of the sustainable development of the country and an important part of the social structure. From a macro point of view, the health management of full-time associate students is the foundation of national sustainable development. Sports nutrition of college students is the key to health management. To a small extent, it is the inevitable choice related to the healthy development of students themselves.

### 1.2. Related Work

The problem of college students' physique has become a serious problem restricting the cultivation of high-quality talents in China, and sports nutrition is the root of college students' low physical quality. In view of the shortcomings of students' physique monitoring platform, Yaman makes full use of the advanced technology of computer and Internet; follows the basic principles of economy, practicality and expansibility, user-friendly, and real-time information exchange; and establishes a college students' physique monitoring and service platform. Through the basic and extended functions of “platform” such as basic assessment, test organization, data management, information release, etc., the expected goals of different levels of teaching management, campus sports, and individual sports intervention of students can be realized, which will have far-reaching practical significance for fitness guidance and exercise [1].

Anxiety or fear associated with physical assessment is defined as social physical anxiety (SPA). Social physical anxiety often occurs in adolescence or early adulthood, and the probability of male and female is equal. A large number of studies have examined this structure, but there is still a gap in the current college students who have both spa and self-efficacy. Therefore, the purpose of Rothberger's research includes quantitative analysis of the relationship among spa, gender, and self-efficacy. Participants included 237 full-time associate students from a university in the southeast who took jogging, body conditioning, or weight training courses. The results of analysis of variance showed that self-efficacy also had significant main effect. The level of spa was higher in those with lower self-efficacy (*P* < 0.001). Stepwise regression analysis showed that self-efficacy and gender were significant predictors of spa. These information can help to formulate intervention measures, reduce the prevalence of spa, and improve the self-efficacy of college students [2].

### 1.3. Innovation

Meta-analysis is the last step of systematic review and the core research method of evidence-based medicine [3]. Its greatest advantages are as follows:

1. By increasing the sample size and reducing the difference caused by random error, the ability of statistical test is improved. It can effectively analyze the relationship between college students' physical health improvement and sports nutrition
2. To explore the heterogeneity of multiple research results, improve the estimation accuracy of effect size, such as whether the research factors provide more accurate effect evaluation for risk factors, solve the inconsistent results of research, and improve the credibility of the conclusion
3. Looking for new hypotheses and research ideas

## 2. The Dynamic Intervention Mechanism of Sports Nutrition Based on the Improvement of College Students' Physical Health

### 2.1. Healthy Physical Fitness

Physical fitness is divided into two parts: healthy fitness and skill fitness. Physical fitness is closely related to health. It refers to cardiovascular function. It is the most ideal performance of lung and muscle. Physical fitness includes the following: cardiorespiratory endurance, muscle strength, body composition, flexibility, and physical fitness. It is also an important benchmark to measure human health. With the growth of age, the health status of the body continues to decline, some body organs will also appear in varying degrees of disease. As a result, health issues are becoming more and more important. The judgment of health performance mainly depends on the appearance, including whether the face is ruddy and tender, whether the skin is dark and yellow, and whether the skin is dull. Although appearance can determine a person's health, it does not mean that they are not ill [4]. With the progress of science and the rapid development of information technology, people pay more and more attention to health. With the appearance of the problem of physical condition, it can provide a reasonable exercise suggestion for people. It can judge whether the body has a certain function through certain tests and then carry out specific exercises in this respect. It is most appropriate to determine the exercise time, intensity, and workload. These indicators can be used as reference [5]. Health and physical fitness can be divided into five categories:

1. Cardiopulmonary endurance: commonly known as aerobic endurance. It is mainly the long-term endurance of long-term exercise of the whole body big muscles. It can reflect the oxygen supply capacity of cells and provide energy for the cardiopulmonary system. Good cardiopulmonary function can effectively improve the ability of oxygen transfer and effectively extend the exercise time
2. Muscle strength and muscle endurance: Muscle state mainly depends on muscle strength and muscle endurance. As muscles are the main body of the body, they are collectively referred to as muscle constitution [6]. Muscle strength refers to the maximum force produced by a group of muscles or muscle groups in the process of contraction, or the maximum resistance that can be overcome. Under specific resistance, the maximum number of times a group of muscles or muscle groups overcome resistance may be an important indicator of an individual's external health
3. Body composition: It refers to the combination ratio of body fat and fat body mass. Body composition mainly refers to the percentage of body fat, including height, weight, and BMI; only a reasonable composition of body composition can keep the body healthy all the time
4. Flexibility and fitness: the stable movement of the main finger joints in the normal range of motion. Flexibility will directly affect the performance of individuals in sports; lack of flexibility will lead to arthritis, hunchback, and back pain and other adverse symptoms
5. Sports developed physical fitness: In addition to the five elements of healthy physical fitness, athletic fitness also includes speed, coordination, sensitivity, reaction time, and explosive force, which are closely related to sports ability

### 2.2. Dietary Behavior of College Students

Breakfast is very important for people's work and study and also an important aspect of keeping healthy. Skipping breakfast or eating breakfast irregularly will bring about various negative consequences. Long time no breakfast incidence in daily life will increase the incidence rate of other diseases, especially the incidence rate of cholesterol disorders, hypoglycemia, and cardiovascular diseases, which can lead to obesity. Breakfast is the easiest to skip between three meals a day, but the nutritional level of breakfast is one-third of the required nutrition [7].

Snacks refer to all kinds of food and drink outside dinner time. Its nutrition and content are much less than a normal meal. If we overeat snacks with low nutritional value and high calorie before lunch, we will lose our appetite for normal diet, lack of food intake, unbalanced nutrition, and even lead to some diseases; the high calorie content of snacks can easily lead to diseases such as high blood pressure and high blood lipids [8]. Most of the snacks students like are puffed food and fried food. Puffed food is a typical food with high oil, high sugar and high calorie, which is three high levels. It is low in nutrients, which can lead to an increase in blood lead levels. Long-term consumption can lead to anemia, epilepsy, and other diseases. Fried food will cause damage to the liver and other body parts; the release of nitrite will cause cancer. All this shows that the harm of snacks cannot be underestimated. The reason why students eat snacks may be hunger caused by lack of food or personal hobbies.

### 2.3. Determination of Weight of Three-Dimensional Health Evaluation Index

Weight is a relative concept for specific indicators. Index weight refers to the relative importance of the index in the overall evaluation, and the weight system should be determined according to the index system [9]. The selection of weight index is actually the process of classifying system rating index. The three-dimensional weight of health evaluation index represents the quantitative distribution of different aspects of the three-dimensional health of the evaluated object, the evaluation process, and the role of each evaluation factor in the overall evaluation. Weight indicators can effectively analyze the relationship between nutrition and physical health. The weight of three-dimensional health evaluation index is the standard to distinguish different three-dimensional health evaluation index, and the three-dimensional weight is reorganized into three-dimensional weight system.

The weight distribution of three-dimensional health assessment index is a typical problem of global crisis, involving many factors. Because the importance of each factor is determined by human subjective judgment, even expert judgment will be affected by some subjective factors. Crisis is inevitable and uncertain [10]. Therefore, in order to improve the reliability of evaluation index weight, it is necessary to find a method to solve the problem of multiple factors. It is more scientific to determine the weight of three-dimensional health evaluation index by AHP. AHP can quantitatively analyze the weight relationship between health evaluation indicators.

Analytic hierarchy process (AHP), also known as analytic hierarchy process (AHP), is a decision-making method which deconstructs the elements of objective decision-making and carries out qualitative and quantitative analysis at the level of standards and schemes [11]. As a decision-making process, it provides a basic method to measure decision-making factors. By making full use of the experience, wisdom, and judgment of experts or collectives and adopting the form of relative scale, quantifiable and nonquantifiable factors are measured. Less quantitative information is used for mathematical calculation and ingestion process decision-making. It provides a simple decision-making method for complex decision-making problems with multiobjective, multicriteria, or unstructured characteristics, which is suitable for situations where it is difficult to directly and accurately measure the decision-making results. In the process of using, the complex problem is decomposed into a hierarchical structure, from the highest level to the lowest level; each level should be compared in pairs to reflect the relative importance of the data sequence. Finally, the overall relative weight of decision-makers' classification is measured by hierarchical relationship.

### 2.4. System Evaluation and Meta-Analysis

Systematic evaluation, also known as “systematic review”, is a new method of literature synthesis proposed by the late epidemiologists in, through comprehensive collection of all relevant randomized controlled trials and scientific quantitative synthesis, so as to obtain comprehensive and reliable conclusions [12]. According to a specific clinical problem, it adopts the principles and methods of clinical epidemiology to reduce bias and random error, systematically and comprehensively collects all published or unpublished clinical research results, selects the literature that meets the quality standards, carries out quantitative analysis or quantitative synthesis, and obtains more reliable conclusions. System evaluation can be qualitative, qualitative system evaluation or quantitative, quantitative system evaluation [13]. Meta-analysis is a kind of systematic evaluation, but systematic evaluation is not always meta-analysis [14].

Sensitivity analysis can reflect the stability of meta-analysis results and is one of the important methods to solve the heterogeneity. This is a method of excluding specific studies and reanalyzing the results of other studies and comparing them with the results before exclusion; stability analysis can be performed on the analyzed results. The robustness of the study and its impact on the comprehensive effect are compared and discussed. Sometimes heterogeneity is caused not only by one study, but also by multiple studies [15]. The heterogeneity test methods are as follows:

(1) $$\begin{array}{c} Q=\sum W_{i}{\left(d_{i}-\bar{d}\right)}^{2}=\sum W_{i}{d_{i}}^{2}-\frac{{\left(\sum W_{i}d_{i}\right)}^{2}}{\sum W_{i}}. \end{array}$$

In the above formula, *W*_i_ is the weight, and the weight of the *i* experiment is calculated according to the following formula:

(2) $$\begin{array}{c} W_{i}=\frac{1}{Var\left(d_{i}\right)}. \end{array}$$

## 3. Experimental Study on the Dynamic Intervention Mechanism of Sports Nutrition Based on the Improvement of College Students' Physical Health

### 3.1. Research Object

This study selects 100 full-time associate students in our university as the research object. According to the needs of the research, before the experiment, the purpose and method of the research should be made clear, so as to ensure the voluntary participation of individuals. Develop a 10-week physical exercise and nutrition intervention program for selected members, and urge them to practice.

### 3.2. Experimental Content

#### 3.2.1. Experimental Grouping

Before the experiment, the subjects' physical condition, physical function, and physical fitness were tested in all aspects. Under the condition that the subjects' physique was basically the same, they were randomly divided into four groups: control group, exercise intervention group, nutrition intervention group, and sports nutrition intervention group, with 25 people in each group. The subjects in the control group did not exercise and did not perform nutrition intervention; the exercise intervention group only exercised without nutritional intervention; the nutrition intervention group only exercised nutritional intervention and no exercise; the exercise nutrition intervention group both exercised and received nutritional intervention.

#### 3.2.2. Test Method

Height refers to the vertical distance from the top of the head to the ground, which reflects the longitudinal extension of the body. It is affected by heredity, sports, nutrition, external environment, race, and other factors, among which the influence of genetic factors is the most obvious. In general, there are significant differences in height between men and women, and there are also significant differences in height development stages between men and women. Generally, girls complete skeletal development at the age of 19-23, while boys finish at the age of 20-24. Height test can be used to understand the physical development of individuals. The normal growth of height at a certain age indicates that growth is good, but the growth of height is slow or stopped, indicating that their development has encountered a bottleneck. Body weight refers to a person's weight. When testing body shape, subjects are required to perform defecation, urination, and other activities before the test and are not allowed to engage in sports activities. Using a height and weight tester, height and weight tests should be done together. Subjects were asked to stand on the tester without shoes and keep their body upright.

Vital capacity refers to the amount of air that a person can exhale with maximum endurance after completing the maximum inhalation of gas, which is a potential manifestation of respiratory function. The size of vital capacity reflects the ability of physical health and is closely related to gender, age and physical condition. In general, electronic vital capacity measuring instrument should be used to test the capacity of vital capacity. During the experiment, the subjects should be asked to inhale as much as possible, and then the instrument should be exhaled as much as possible until it cannot be exhaled. The maximum value of the experimental results should be obtained after three experiments.

In the 800-meter experiment, at least two people were tested in pairs from the beginning. When they heard the “run” command, the subjects began to run. The timekeeper saw the flag shaking and began timing when the subject's torso reached the vertical horizontal finish line. Before the 800-m test, standard timer shall be used for calibration, and the error shall not exceed 0.3 s/min. The standard timer is selected according to Beijing time, and the error is less than 0.5 s/h. Record test results in minutes and seconds, excluding decimal points.

Nutrition intervention is divided into two parts: nutrition education and food program. Nutrition education is mainly to train and disseminate nutrition knowledge to the subjects before and during the experiment and to send out questionnaires to the subjects, so as to understand their understanding of nutrition knowledge. Before and after the intervention, professional nutritionists should give lectures on nutrition related knowledge and then conduct a questionnaire survey on the subjects again to test the same subjects. The lecture mainly focuses on the problems found in reasonable diet and nutrition research and provides guidance for those who have problems. Food supplements are formulated under the guidance of doctors and nutritionists. Food supplements determine the type of food and the amount of food that people must eat every day, as well as the vitamins and proteins that people need to supplement every day. As for the problem of insufficient intake of some substances, it is necessary to adjust the food according to individual conditions. At the same time, parents and teachers are required to help and supervise the experiment. During the implementation of the nutrition intervention program, food supplement makers should visit the school regularly to check the nutritional status of students and solve relevant problems.

### 3.3. Mathematical Statistics

Use statistical software to input data and statistics. Statistical software is divided into data statistics and statistical analysis software. In this paper, Matlab software is used for data statistics. Firstly, the mean and standard deviation of the differences between the experimental group and the control group before and after the intervention were calculated. According to the types given in the systematic assessment and meta-analysis, the differences before and after the intervention and the differences before and after the intervention were calculated. The weighted average difference of each physical state index is taken as the effect scale. The statistical results should include the comprehensive effect size and the confidence interval.

## 4. Experimental Analysis on the Dynamic Intervention Mechanism of Sports Nutrition for Improving College Students' Physical Health

### 4.1. Analysis on the Dynamic Change of College Students' Physique Grade from 2017 to 2019

Talent competition is the theme of future social competition. As the main force of the country's future construction, students must have strong character in addition to noble morality and profound knowledge. In order to objectively and accurately reflect the dynamic changes of students' physical development, this study obtained the physical health level report of male and female students in our school from 2017 to 2019. According to the national students' physical health standard, a comprehensive evaluation of college students' physical condition is carried out, which is defined as follows: *x* < 60 points: fail; 60 ≤ *x* < 70: pass; 70 ≤ *x* < 85: good; and *X* ≥ 85: excellent. The evaluation results are shown in Table 1.

From the data in the table, it can be seen that in these three years, college students' physique has developed in many ways. From the perspective of male students' physique, the proportion of excellent physique of male students in our school accounted for 0.21, 0.24, and 0.26, respectively, in three years, while the proportion of good physique hovered between 0.34 and 0.39, and the proportion of failed students showed a trend of first rising and then declining, and the overall physical fitness level of boys was developing in a good direction. In terms of female students' physique, the overall trend of female students' physique is declining. Although the proportion of excellent students is 0.13 in the past three years, the proportion of good and qualified students has been declining slowly, and the proportion of failing to pass has increased from 0.11 to 0.24. In order to better understand the physical condition of contemporary college students, the results of physical fitness grade of our college students in 2019 are selected to make a histogram, as shown in Figure 1.

From the data in the figure, it can be seen that the number of boys with excellent physique is nearly three times higher than that of girls. Although there are also reasons for the large number of boys, it is undeniable that the physique of boys is better than that of girls from the data. The number of students with good constitution is higher than that of female students. The physique grades of female students are mainly good and pass, and the number of students who fail is also too much. Generally speaking, boys' physical performance is OK, and they need to continue to refuel, while girls' physique is relatively weak, so they need to strengthen physical exercise and nutrition supply.

### 4.2. Changes in Body Mass Index

Before the experiment, the body shape indexes of the control group, the exercise group, the nutrition group, and the sports nutrition group were tested. The test results show that there is no significant difference in the body shape indexes of the four groups of students, which indicates that the body shape indexes of the students are basically consistent, which can also ensure that the deviation of the experimental objects is small, and the experimental data is relatively reliable.

As shown in Figure 2, there is no significant difference in height index between the control group, the nutrition group, and the nutritional exercise group. It can be seen that nutrition and sports have little effect on the height level of college students. The main reason is that the height of college students is affected by related factors and environmental factors.

In terms of body weight, compared with the control group, the exercise group and the nutritional exercise group decreased significantly after the experiment. Compared with the exercise group, the body weight of the nutrition group increased significantly after the experiment. The experiment shows that scientific nutrition and physical exercise can help to lose weight, but unilateral nutrition control and physical exercise cannot achieve good results. This is mainly due to the individual in the experimental process to maintain a certain amount of exercise and reasonable diet. When the human body has just done sports activities, weight loss effect is obvious. This is because you consume a lot of water and fat during exercise, and then it slows down. In terms of energy supply, the intervention program designed in this study maintained the heart rate of subjects at 130 beats/min, and then even reached 160 beats/min, which is equivalent to the speed of 3 km per hour for long-distance running. This intensity of long-distance running speed is in the range of air energy supply, energy consumption is mainly provided by fat decomposition, so everyone's weight has different degrees of decline, which can also provide scientific theoretical basis for obese people to take weight loss measures.

### 4.3. Changes in Vital Capacity and Body Mass Index

Vital capacity body mass index mainly reflects the correlation between lung capacity and body weight through the ratio of lung capacity to body weight and the relative value of lung capacity per kilogram of body weight. It is used for objective quantitative comparative analysis of individuals and groups of different ages and genders. It can be used for reference in the selection of athletes and the comprehensive evaluation of students' physique. The calculation formula is: vital capacity/body weight, the unit of measurement is vital capacity in ml and body weight in kg.

As shown in Figure 3, compared with the control group, the vital capacity of the exercise group was significantly increased. Compared with exercise group and diet group, the survival ability of exercise group was significantly improved. After nutrition intervention, the individual vitality was enhanced, and the exercise group and exercise nutrition group increased significantly, which indicated that physical exercise can increase the lung capacity of college students. The size of vital capacity is closely related to exercise intensity. With the increase of exercise intensity, lung capacity will also increase. Under the effect of exercise plan, individuals carry out long-term moderate intensity exercise, and the body produces a lot of carbon dioxide while generating energy. Carbon dioxide is excluded from the body, which requires the respiratory system to increase workload in the body, increase the depth of breathing, exercise respiratory muscle groups, and increase the strength of respiratory muscles. With the extension of exercise time, the respiratory rate will also decrease, showing a slow and deep state. This situation may also lead to respiratory muscles fully rest in the process of ensuring lung aerobic, effectively increase the breathing capacity, thus increasing the vital capacity, so as to make individuals less prone to asthma during exercise.

Specific diet can also increase the lung capacity of college students. Eating certain vegetables and fruits does help people breathe more freely. Apples and tomatoes are especially useful for increasing lung capacity. Compared with the data of nutrition group and sports group, physical exercise can improve the vitality of college students more than nutrition intervention. In this regard, the comprehensive intervention of sports intervention and nutrition intervention has a more significant impact on college students' lung capacity. Lack of exercise is also the main reason for low lung capacity, especially in endurance sports such as long-distance running. At the same time, due to the existence of various objective reasons, such as heavy schoolwork burden and less spare time, they seldom take part in physical exercise.

### 4.4. Changes in Physical Fitness of Subjects

Exercise has an important impact on the explosive power of lower limbs, and nutrition intervention combined with exercise can improve the explosive power of lower limbs more obviously. Both the exercise group and the exercise nutrition intervention group improved the explosive strength of lower limbs and the level of body coordination. Nutrition intervention group had no effect on the explosive power of lower limbs and individual body coordination. In the 800-meter running experiment, there was no significant difference in the control group before and after the experiment, the difference was significant in the exercise group, there was no significant difference in the nutrition group before and after the experiment, but there was a very significant difference in the sports nutrition group before and after the experiment. The experiment shows that exercise has an important influence on the improvement of endurance quality. In the process of combining nutrition intervention with exercise, the improvement of endurance quality is more obvious, and simple nutrition does not improve the aerobic endurance performance of subjects, as shown in Figure 4.

The intervention plan has fundamentally promoted the physical health of college students. Reasonable sports content is helpful to enhance college students' physique. Therefore, in the physical education teaching, teachers must adjust the logical content and method of teaching according to the students' physical conditions so that students can make full use of the opportunities of classroom exercise, especially to improve the upper limb strength, lower limb strength, flexibility, and other qualities, and should arrange teaching items.

## 5. Conclusion

Adults who do not exercise much on a daily basis are usually in poor physical condition and are prone to cardiovascular disease. Participating in more sports and planning a healthy and nutritious diet can effectively improve physical fitness. Exercise intervention can effectively prevent adult chronic diseases caused by unhealthy lifestyle. Under the joint action of genetic and environmental factors, the static lifestyle in childhood can lead to obesity and various metabolic diseases in adulthood. If the number of activities is less than this limit, it will lead to osteoporosis, cardiovascular disease, and premature death. If the exercise habit is formed from childhood, it will prolong the life span and have a beneficial effect on the body.

When making exercise intervention plan, it is important to consider the characteristics of different students and teach students according to their aptitude. Physical education classroom management in colleges and universities should be closely combined with teaching practice and management principles. School teaching, sports content, reasonable arrangement of sports facilities, and sports courses fully mobilize the enthusiasm of teachers and students for sports learning. In order to improve the students' comprehensive quality, we must realize the comprehensive development of morality, intelligence, and physique, establish a good teaching mode, and attach importance to students' physical fitness test. Physical condition test can directly reflect the current physical condition. The results of physical test are analyzed according to different data and contents. Physical education teaching is designed according to students' physical health condition, which truly serves students and improves their physical health level.

The importance of young people's daily intake of nutrients needs to be strengthened. Consciousness often determines action, and college students' awareness of participating in physical exercise is weak. Therefore, in physical education, teachers should convey to students the value that physical exercise is beneficial to the body and health, so as to improve the physical fitness and health awareness of college students. Because school meals may not meet the nutritional needs of full-time associate students for one day, regular lectures on nutrition and physical exercise knowledge are held to improve students' understanding of nutrition and sports, so as to timely supplement the nutrition required by human body.

## Figures and Tables

**Figure 1:** The dynamic change of students' constitution grade in our university.

**Figure 2:** Body mass index changes.

**Figure 3:** Changes of vital capacity and body mass index.

**Figure 4:** 800 meter running time.

**Table 1:** Physical fitness grade of college students in 2017-2019.

	Year	Excellent		Good		Pass	
		Number of people	Proportion	Number of people	Proportion	Number of people	Proportion
Boys	2017	463	0.21	843	0.39	654	0.31
	2018	582	0.24	831	0.34	731	0.3
	2019	710	0.26	1083	0.39	732	0.26
Girls	2017	185	0.13	539	0.37	564	0.39
	2018	223	0.13	621	0.37	501	0.3
	2019	259	0.13	703	0.35	568	0.28

## Data Availability

No data were used to support this study.
